# Detection of Cardiovascular Disease Based on PPG Signals Using Machine Learning with Cloud Computing

**DOI:** 10.1155/2022/1672677

**Published:** 2022-08-04

**Authors:** Tariq Sadad, Syed Ahmad Chan Bukhari, Asim Munir, Anwar Ghani, Ahmed M. El-Sherbeeny, Hafiz Tayyab Rauf

**Affiliations:** ^1^Department of Computer Science and Software Engineering, International Islamic University Islamabad, Pakistan; ^2^Division of Computer Science, Mathematics and Science, Collins College of Professional Studies, St. Johns University, New York 11439, NY, USA; ^3^Industrial Engineering Department, College of Engineering, King Saud University, P.O. Box 800, Riyadh 11421, Saudi Arabia; ^4^Centre for Smart Systems, AI and Cybersecurity, Staffordshire University, Stoke-on-Trent, UK

## Abstract

Hypertension is the main cause of blood pressure (BP), which further causes various cardiovascular diseases (CVDs). The recent COVID-19 pandemic raised the burden on the healthcare system and also limits the resources to these patients only. The treatment of chronic patients, especially those who suffer from CVD, has fallen behind, resulting in increased deaths from CVD around the world. Regular monitoring of BP is crucial to prevent CVDs as it can be controlled and diagnosed through constant monitoring. To find an effective and convenient procedure for the early diagnosis of CVDs, photoplethysmography (PPG) is recognized as a low-cost technology. Through PPG technology, various cardiovascular parameters, including blood pressure, heart rate, blood oxygen saturation, etc., are detected. Merging the healthcare domain with information technology (IT) is a demanding area to reduce the rehospitalization of CVD patients. In the proposed model, PPG signals from the Internet of things (IoT)-enabled wearable patient monitoring (WPM) devices are used to monitor the heart rate (HR), etc., of the patients remotely. This article investigates various machine learning techniques such as decision tree (DT), naïve Bayes (NB), and support vector machine (SVM) and the deep learning model one-dimensional convolutional neural network-long short-term memory (1D CNN-LSTM) to develop a system that assists physicians during continuous monitoring, which achieved an accuracy of 99.5% using PPG-BP data set. The proposed system provides cost-effective, efficient, and fully connected monitoring systems for cardiac patients.

## 1. Introduction

Healthcare is one of the most important domains that need faster development. Currently, digital health has gradually increased in our daily life through wearable medical devices such as smartwatches and smartphone applications for real-time monitoring and diagnostic purpose [1]. The innovation of wireless communication technology and the availability of electronic components enabled the Internet of things (IoT) application [2] in wearable patient monitoring (WPM) devices.

Such models specify that this is a small addition in the field of artificial intelligence, robotics, and telemedicine [1]. The IoT in the health sector will probably reach around 409.9 billion USD in 2022 according to Grand View Research Inc. [3]. A variety of WMP devices are available that use a wireless network to transmit medical information to mobile and Web applications, but they face accuracy, precision, and reliability issues [4]. Hypertension is the important risk factor of cardiovascular diseases (CVDs) [5]; according to the report of the World Health Organization (WHO), CVD is the main chronic disease and the major contribution to the global burden of diseases. The report states that 31% of the deaths around the world are caused by CVD [6]. Thus, blood pressure (BP) can be monitored for the primary detection of CVD. Three parameters are mostly evaluated, such as systolic blood pressure (SBP), diastolic blood pressure (DBP), and mean arterial pressure (MAP), to find BP in millimeters of mercury (mmHg) [7, 8]. Two common ways are used for finding BP: noninvasive and invasive methods. Noninvasive BP measurement is done through cuff-based readings, but it is not comfortable for infants, injured, and overweight people [9]. Also, its end result is discrete (that is, some set of intervals is required) and thus uncomfortable to the patient. The invasive procedure involves arterial lines management for monitoring continuous BP, but it is not appropriate to employ due to vulnerability of infections [10]. In cardiology, patients' home is preferred for continuous monitoring of temperature, blood pressure, heart rate, and ECG of the patients. Thus, a cuff-less, noninvasive, and continuous BP monitoring system is required.

### 1.1. Calculating BP through Photoplethysmography

Photoplethysmography (PPG) has been innovated to monitor BP without a need of an inflatable cuff [11, 12]. PPG is a versatile and low-cost technology [9], and it uses human skin vessels to find changes in light transmitted or reflected through the photoelectric sensor [13]. It signifies the variation of human blood volume and differentiates the systolic and diastolic processes of the heart, which are associated with BP. The light emitting diode (LED) and photodiode (PD) are used to evaluate the variations in the reflected light. Moreover, the estimation of BP using PPG is very authentic. PPG can be extended to different aspects of cardiovascular surveillance, including identification of blood oxygen saturation, heart rate, BP estimation, cardiac output, respiration, arterial aging, endothelial control, microvascular blood flow, and autonomic function. PPG does not need any certain method to connect sensors at predefined locations in the body [14]; simply, it can be collected from the wrist, finger, or earlobe [15]. This simplicity has made PPG an eye-catching biosignal usually for wearable applications to estimate heart rate (HR) during exercise and other physical movements.

The sample of PPG signal captured and its sinusoidal waves is illustrated in Figures 1 and 2, respectively.

Various methods such as periodograms, spectrograms, and wavelets are used to evaluate the biosignals as demonstrated in Figures 3–5, respectively.

### 1.2. Motivation

High BP puts strain on the heart and the arteries, increasing the probability of heart attack, dementia, stroke, and kidney diseases. Continuous monitoring is crucial to control and manage high BP. Moreover, various researchers show that home-based noninvasive sensors can be deployed for remote monitoring to reduce rehospitalization of cardiac patients [16]. Like other computing systems, the WPM devices have hardware and software modules. Hardware is concerned with data collection, conversion of electrical signals, and communication with the decision-making subsystem. Software is the second module concerned with making decisions based on the obtained signals. The second module is the main focus where machine learning becomes useful. The advancement in the field of machine learning is probably increasing the diagnostic prediction through WPM devices. Thus, it is unavoidable that machine learning techniques are required to improve the reliable diagnosis of different diseases.

### 1.3. Article Contributions

The proposed work is used to monitor cardiac disorder with the help of WPM devices, cloud computing, and artificial intelligence (AI). The main contributions of this manuscript are as follow:

- A novel framework has been proposed to deal with challenges of integration of remote patient data from different sources and make an accurate diagnosis.
- The proposed CAD system receives PPG-recorded signals using IoT-enabled WPM and performs intelligent diagnostic process with significantly improved accuracy.
- To meet the excessive resources requirement of intelligent algorithms on the medical data, the proposed framework uses cloud computing.
- The proposed framework ensures timely diagnoses along with doctor's recommendation to the concerned patient in an effective manner.

### 1.4. Article Layout

The rest of the paper is structured in the following sequence: Section 2 provides a brief description of the related literature; Section 3 describes the proposed method; results and discussions are reported in Section 4, and the conclusion and future direction are presented in Section 5.

## 2. Related Literature

A rapid growth in the adoption of WPM and Internet of things (IoT) models around the world has been observed over the last decades. Advancement in the e-healthcare systems and smart home automation technologies provide the facility to avail in-home medical services without hospital visits. Thus, the IoT has been recognized as a possible solution to relieve the burdens on healthcare societies. Various researchers and foundations proposed different models in the field of e-health, remote healthcare, and smart healthcare system [17–19]. An extensive work of IoT in healthcare applications is carried out in [20] with emphasis on problems and their possible solutions.

Automation for smart home is an emerging domain of IoT and has been applied in several areas to assist in daily living to support humans and to make their life easy; for example, home appliances based on remote control [21], energy management in the house [22], security systems [23], movement detection in the home [24], and providing healthcare facility to disabled, outdoor patients, and elderly persons [25, 26].

Agarwal and Lau [27] proposed a health monitoring system to evaluate the blood pressure (BP) of patients using smart devices. They argued that the recorded values of systolic and diastolic pressure can be easily forwarded to a cardiologist or physician through a Web interface that can further be evaluated by a physician to facilitate the patient online. A healthcare system employing body sensor network (BSN) has been proposed by Gope and Hwang [28]. The proposed system also called BSN-Care is used to measure the physiological parameters BP and electrocardiogram (ECG) to check heart condition through a WPM device. The data received from the patient's body are sent to the BSN-Care server and then are used for evaluation. In case of abnormality, the system alerts the family member and physician of the patient for a prompt response.

Chen et al. [29] recommended an e-healthcare system via an RFID system. The system is used to evaluate the patients' health condition and performs communication between the doctor and the patient. It can also be employed to collect patients' information such as temperature and BP through BSN. Furthermore, it is also capable to maintain the medical history and profile of the patients for future use. Chatrati et al. [30] developed a health monitoring system based on a smart home for remote monitoring of chronic patients related to BP and diabetes. The system is utilized to monitor the patient's BP and glucose level from home and send alerts and real-time notifications to registered healthcare centers or physicians in case of any abnormality. Xiao et al. [31] employed a model based on compressed sensing for recognition of PPG signals, where the authors applied the discrete wavelet transform as features extraction followed by SVM classifier and attained an accuracy of 91.31%.

## 3. Proposed Method

It is dangerous to provide patient services physically during the COVID-19 pandemic; hence, online consultation and telemedicine are becoming more popular. The number of CVD patients is increasing day by day, causing more deaths, and is further multiplied during the current pandemic. To prevent this increasing number and reduce the burden on the healthcare society, constant monitoring of CVD patients is required. Despite the advancement of diagnostic procedures in CVDs, main clinical issues persist in this area. Integrating data from different sources for remote patients and making a proper diagnosis is a major challenge. Machine learning has usually been costly and performed by scientists through high-performance processors. As we know that professional processing units are too costly, machine learning can be accomplished through cloud environments [32, 33]. This article proposes a cloud-based CVD diagnosis system to facilitate the assessment and monitoring of patients remotely. In this model, we focused to diagnose cardiac diseases such as normal, prehypertension, stage 1 hypertension, and stage 2 hypertension.

In the proposed method, the PPG signals are recorded through IoT-enabled WPM devices during physical activity such as low-, medium-, and high-intensity arm movements containing driving, walking, and sitting for a while to find heart rates.

The PPG signals are then sent through the Internet to the CAD server in the cloud for further processing. The diagnostic report is sent back to the concerned patient via the doctor's recommendation for a better prescription to the patients, after processing through machine learning algorithms configured in the cloud. The overall framework of the proposed system is exhibited in Figure 6, containing WPM and cloud-based CAD server. Using such a system, patients would be capable to accomplish the goals of CVD diagnosis at home at a minimal cost.

### 3.1. PPG-BP Data Set

In this work, we used an openly accessible data set called PPG-BP [34], which is a combination of PPG and BP. This database incorporates the comprehensive clinical and anonymous data of patients admitted to Guilin People's Hospital, China. The clarity of the data permits clinical analyses to investigate and enhance the understanding of connections between PPG signals and cardiovascular health. Moreover, the goal is to provide an effective, simple, and noninvasive technology such as easy to employ and wearable. The PPG-BP data set was gathered from 219 patients, aged between 21 and 86 years. 48% of the data were of males. The data set comprises various diseases, including BP, HR, hypertension, etc., as presented in Table 1. In this dataset, the outcome of the data is categorized into four labels, i.e., Prehypertension, Stage 2 Hypertension, Stage 1 Hypertension, and Normal. Most of the data in this dataset contain the category of Prehypertension and Normal labels as illustrated in Figure 7.

### 3.2. PPG-DaLiA Data Set

In this work, we used an openly accessible data set called PPG-DaLiA, i.e., PPG data set for motion compensation and heart rate estimation in daily life activities [30]. The activities and their duration included in the data set are presented in Table 2. This data set contains eight different types of activities, which are usually performed in daily routine. The activities included low-, medium-, and high-intensity arm movements such as driving, walking, and table soccer, respectively, to find variable heart rates. Figures 8 and 9 demonstrate the heart rate information extracted from the ECG signal during sequence of activites performed by two different persons.

### 3.3. Automatic Detection of Heart Rate

In order to thoroughly evaluate the abundant information contained in the PPG signals, it is essential to acquire the most reliable and high-quality PPG signal. Moreover, we must ensure that the obtained data have complete heartbeat, less noise, cycles, and motion artifacts. The above two mentioned data sets are used for heart rate detection. The PPG-BP data set is evaluated through the conventional method of machine learning, and the second data set called PPG-DaLiA is evaluated through one-dimensional convolutional neural network-long short-term memory (1D CNN-LSTM).

### 3.4. Detection of Heart Rate through Machine Learning

The PPG-BP data set contained all the said information. Such data can be evaluated through different machine learning algorithms with different parameters. Supervised machine learning classifiers such as decision tree (DT), naïve Bayes (NB), support vector machine (SVM), and ensemble classifiers are used to evaluate the proposed model using k-fold cross-validation [35].

#### 3.4.1. Decision Tree (DT)

DT classifies the instances by arranging them based on values via a top-down approach [36]. The variable used in a splitting condition is chosen according to the splitting criteria to reduce impurity. To select the best value, we used the Gini diversity index (GDI) as a splitting condition, which is formulated as in equation (1):

(1) $$\begin{array}{c} x\left(t\right)=\sum_{y\neq x}P\left(y|t\right)P\left(x|t\right). \end{array}$$

The GDI is the probability of misclassification; thus, the efficiency of GDI is to perform the split at a node where the probability of misclassification is lower. The parameters employed during the experiment are presented in Table 3.

#### 3.4.2. Ensemble Classifier

An ensemble classifier involves multiple learning approaches such as boosting and bagging to achieve better performance. During the experiments using the ensemble classifier, the proposed approach achieved the highest results. The parameters used for this classifier are presented in Table 4.

### 3.5. Detection of Heart Rate through 1D CNN-LSTM

The deep learning models are applied in many real-world applications [37]. In this section, we applied the 1D CNN-LSTM model for heart rate detection using the PPG-DaLiA data set. The 1D CNN can be used to extract robust features of 1D time-series sequence data using convolution operations through several filters. In this work, the 1D CNN-LSTM model contains two convolution layers, one LSTM layer, two fully connected (FC) layers, and a soft-max output layer, as illustrated in Figure 10.

### 3.6. Performance Evaluation

The performance of the proposed model has been evaluated using accuracy, confusion matrix, and ROC curve. The confusion matrix is used to evaluate parameters such as TP (true positive), TN (true negative), FP (false positive), and FN (false negative). Moreover, the ROC curve is employed to evaluate the classification performance through graphical portrayal [38]. The ROC curve is computed by drawing false positive rate (FPR) against true positive rate (TPR) [39].

## 4. Results and Discussion

To evaluate the performance of classification, results obtained using parameters like accuracy, confusion matrix, and ROC curve are used. The obtained accuracy using the PPG-BP data set is presented in Table 5. It shows that all types of decision trees (fine, medium, and coarse) achieved the highest results of 99.5%. Similarly, the ensemble classifier (bagged tree) achieved the second highest result of 97.7%. These results obtained through a decision tree and ensemble classifier are further assessed through confusion matrix, as presented in Figures 11 and 12, respectively.

The ROC curve is also used to exhibit the analysis results achieved through the best classifier.  Figure 13 demonstrates the decision tree classification performance with an AUC value of 1.00, while Figure 14 shows the performance of ensemble classifier (bagged trees) with an AUC value of 0.99.

Similarly, to evaluate the classification performance of PPG-DaLiA data set using the 1D CNN-LSTM model, an 80-20% split is used to train the model using 50 epochs. The proposed approach, in this case, has achieved an accuracy of 97.56%. The result is further evaluated through confusion matrix, as presented in Figure 15. It is clear from both data sets that we achieved better accuracy using the PPG-BP data set through conventional methods of learning compared with PPG-DaLiA data set. The reason is that the PPG-DaLiA data set is complex, although the model is trained using an advanced deep learning method. However, this result can be further improved using a hyperparameter setting.

Furthermore, some key challenges are also concern with machine learning and deep learning models in CVD diagnosis. For example, any wrong classification might produce severe damage and bad impact.

### 4.1. Comparison with Existing Work

The proposed technique is also compared with some recent work, as presented in Table 6. In Table 6, it is clearly indicated that our proposed technique is better in terms of accuracy compared with [40]. However, the accuracy obtained in [41] is equal to the proposed one, and hence we added another data set and applied deep learning in the proposed work to gain more attraction.

## 5. Conclusions and Future Work

This research work employed machine learning and deep learning to analyze CVD patients using PPG signals. The proposed system was evaluated through various models on publicly available data sets such as PPG-BP and PPG-DaLiA data sets. The proposed model achieved an accuracy of 99.5% and 97.56% using the PPG-BP and PPG-DaLiA data sets, respectively. The reason for choosing PPG signal in the proposed work is that it is a low-cost technology, which can easily be captured through IoT-based WPM devices and be processed on cloud computing. The employment of such a model is very helpful for the community, especially the people residing in remote and backward areas. In the future, this work may focus on more data sets with the involvement of image processing and advanced deep learning methods.

The notations that are used in this paper are summarized in Table 7.

## Figures and Tables

**Figure 1:** PPG signal.

**Figure 2:** PPG sinusoidal waves.

**Figure 3:** Periodograms.

**Figure 4:** Spectrograms.

**Figure 5:** Wavelets.

**Figure 6:** Proposed method.

**Figure 7:** Data distribution based on hypertension.

**Figure 8:** Heart rate information extracted from person 1.

**Figure 9:** Heart rate information extracted from person 2.

**Figure 10:** Illustration of 1D CNN-LSTM.

**Figure 11:** Confusion matrix through decision tree using PPG-BP data set.

**Figure 12:** Confusion matrix through ensemble classifier (bagged trees) using PPG-BP data set.

**Figure 13:** ROC curve: decision tree.

**Figure 14:** ROC curve: ensemble classifier.

**Figure 15:** Confusion matrix through 1D CNN-LSTM model using PPG-DaLiA data set.

**Table 1:** PPG-PB data set.

	Subject_ID	Sex (M/F)	Age (year)	Height (cm)	Weight (kg)	Systolic BP (mmHg)	Diastolic BP (mmHg)	Heart rate (b/m)	BHI (kg/m^2^)	Hypertension
0	2	Female	45	152	63	161	89	97	27.27	Stage 2 hypertension
1	3	Female	50	157	50	160	93	76	20.28	Stage 2 hypertension
2	6	Female	47	150	47	101	71	79	20.29	Normal
3	8	Male	45	172	65	136	93	87	21.97	Prehypertension
4	9	Female	46	155	65	123	73	73	27.06	Prehypertension
…	⋯	⋯	⋯	⋯	⋯	⋯	⋯	⋯	⋯	⋯
214	415	Male	24	180	70	111	70	77	21.60	Normal
215	416	Female	25	156	47	93	57	79	19.31	Normal
216	417	Male	25	176	55	120	69	72	17.76	Stage 2 prehypertension
217	418	Male	25	173	63	106	69	67	21.05	Normal
218	419	Male	24	175	58	108	68	65	18.94	Normal

**Table 2:** Activities with duration.

S/No.	Activities	Duration
1	Sitting	10
2	Stairs	5
3	Table soccer	5
4	Cycling	8
5	Driving	15
6	Launch	30
7	Walking	10
8	Working	20

**Table 3:** Parameters used for decision tree.

Classifier	Type	Split criteria	Max no. of splits
Decision tree	Fine	GDI	100
	Medium		20
	Coarse		4

**Table 4:** Parameters used for ensemble classifier.

Type of ensemble	Learner	No. of learners
Bagged trees	Decision tree	30

**Table 5:** Obtained accuracy using PPG-BP data set.

Data set	Classifier	Type	Accuracy (%)
PPG-BP	Decision tree	Fine tree	99.5
		Medium tree	99.5
		Coarse tree	99.5
	Naïve Bayes	Gaussian naïve Bayes	90.4
		Kernel naïve Bayes	87.2
	SVM	Linear SVM	94.1
		Quadratic SVM	88.6
		Cubic SVM	87.2
		Fine Gaussian SVM	49.3
		Medium Gaussian SVM	83.6
		Coarse Gaussian SVM	74.4

**Table 6:** Comparison with published work.

Ref.	Method	Data set	Accuracy (%)
Yen et al. [40]	ResNetCNN	PPG-BP	73
Nour and Polat [41]	Decision tree	PPG-BP	99.5
Proposed	Decision tree	PPG-BP	99.5
Proposed	CNN-LSTM	PPG-DaLiA	97.56

**Table 7:** Summary of the notation.

Notation	Meaning
BP	Blood pressure
CAD	Computer aided diagnosis
CVD	Cardiovascular disease
DBP	Diastolic blood pressure
DT	Decision tree
ECG	Electrocardiogram
FN	False negative
FP	False positive
FPR	False positive rate
HR	Heart rate
IoT	Internet of things
LED	Light emitting diode
NB	Naïve Bayes
PD	Photodiode
PPG	Photoplethysmography
SVM	Support vector machine
SBP	Systolic blood pressure
TN	True negative
TP	True positive
TPR	True positive rate
SBP	Systolic blood pressure
SBP	Systolic blood pressure
WHO	World Health Organization

## Data Availability

In this work, we used publicly available data sets called PPG-BP [34] to analyze the clinical data and PPG-DaLiA dataset [30] to evaluate motion compensation and heart rate estimation in daily life activities.
